The article "Functional Expression of Human α9* Nicotinic Acetylcholine Receptors in X. laevis Oocytes Is Dependent on the α9 Subunit 5′ UTR" was published in 2013. Journal: PLoS One.

# Functional Expression of Human α9* Nicotinic Acetylcholine Receptors in *X. laevis* Oocytes Is Dependent on the α9 Subunit 5′ UTR

**DOI:** 10.1371/journal.pone.0064655

**Published:** 2013-05-22

**Authors:** Olena Filchakova, J. Michael McIntosh

**Affiliations:** 1 Interdepartmental Program in Neuroscience, University of Utah, Salt Lake City, Utah, United States of America; 2 George E. Wahlen Veterans Affairs Medical Center, Salt Lake City, Utah, United States of America; 3 Department of Psychiatry, University of Utah, Salt Lake City, Utah, United States of America; 4 Department of Biology, University of Utah, Salt Lake City, Utah, United States of America; Weizmann Institute of Science, Israel

## Abstract

Nicotinic acetylcholine receptors (nAChRs) containing the α9 subunit are expressed in a wide variety of non-neuronal tissues ranging from immune cells to breast carcinomas. The α9 subunit is able to assemble into a functional homomeric nAChR and also co-assemble with the α10 subunit into functional heteromeric nAChRs. Despite the increasing awareness of the important roles of this subunit in vertebrates, the study of human α9-containing nAChRs has been severely limited by difficulties in its expression in heterologous systems. In *Xenopus laevis* oocytes, functional expression of human α9α10 nAChRs is very low compared to that of rat α9α10 nAChRs. When oocytes were co-injected with cRNA of α9 and α10 subunits of human *versus* those of rat, oocytes with the rat α9 human α10 combination had an ∼-fold higher level of acetylcholine-gated currents (I_ACh_) than those with the human α9 rat α10 combination, suggesting difficulties with human α9 expression. When the ratio of injected human α9 cRNA to human α10 cRNA was increased from 1∶1 to 5∶1, I_ACh_ increased 36-fold (from 142±23 nA to 5171±748 nA). Functional expression of human α9-containing receptors in oocytes was markedly improved by appending the 5′-untranslated region of alfalfa mosaic virus RNA4 to the 5′-leader sequence of the α9 subunit cRNA. This increased the functional expression of homomeric human α9 receptors by 70-fold (from 7±1 nA to 475±158 nA) and of human α9α10 heteromeric receptors by 80-fold (from 113±62 nA to 9192±1137 nA). These findings indicate the importance of the composition of the 5′ untranslated leader sequence for expression of α9-containing nAChRs.

## Introduction

Nicotinic acetylcholine receptors (nAChRs) are ACh-gated ion channels implicated in many physiological as well as pathophysiological processes. The role of nAChRs in mediating EPSPs at synapses in autonomic ganglia [1], [2] and at the skeletal neuromuscular junction is well established [3], [4]. In the CNS, nAChRs are involved in modulation of neurotransmitter release [5] and in attention and memory [6], [7]. The pathological conditions where involvement of nAChRs have been implicated include Alzheimer's and Parkinson's diseases [8], [9], nicotine addiction [10], [11] and schizophrenia [12], [13]. Seventeen vertebrate nAChR subunits have been cloned to date (α1 through α10, β1 through β4, γ, δ, and ε) [14]. The nAChR is formed from five subunits, either homomeric receptors (α7, α9) containing five identical subunits or heteromeric receptors (for example, α4β2, α3α5β4, α6α4β2β3, or α9α10).

α9-containing nAChRs are unique among neuronal nAChRs in that they are found mainly outside of the CNS [15], [16], [17], [18], [19]. Also, unlike other nAChRs, they are inhibited by nicotine [15], [20], [21]. α9-containing nAChRs play roles in pain [22], [23], [24], [25], [26], [27], inflammation, keratinocyte adhesion [28], and in mediating synaptic transmission between the efferent olivocochlear fibers and cochlear hair cells [29], [30].

The article "Functional Expression of Human α9* Nicotinic Acetylcholine Receptors in X. laevis Oocytes Is Dependent on the α9 Subunit 5′ UTR" was published in 2013. Journal: PLoS One.

With advances in molecular biology, it became possible to isolate and sequence the genes encoding nAChRs. α9 and α10 subunits were among the last nicotinic receptor subunits to be isolated and characterized. The clone encoding the α9 subunit was originally obtained from a rat olfactory epithelium cDNA library [15]. *X. laevis* oocytes injected solely with rat α9 cRNA yielded homomeric receptors that responded to 100 µM ACh with currents that ranged from 20 to 500 nA [15]. The clone encoding the rat α10 subunit was isolated from an adult rat cochlea cDNA library [31]. The coinjection of rat α9 and rat α10 cRNAs into oocytes resulted in oocytes with ∼100-fold larger ACh-gated currents (I_ACh_) than oocytes injected solely with α9 cRNA. Subsequently, the sequences of human α9 and α10 subunits were determined from keratinocytes [28] and inner-ear neuroepithelium [32], respectively.

To study the pharmacological properties of nAChRs, heterologous expression systems are often used. Mammalian cell lines such as HEK293 and SH-EP1 cells are frequently used to characterize nAChRs [33], [34]. Besides mammalian cells, oocytes of *Xenopus laevis*, the African clawed frog, have been frequently used for heterologous expression. These oocytes provide several advantages for the study of receptors. They are large and thus easy to handle and to inject with RNA, have long life-times (several days) and can be maintained under relatively simple culture conditions. Oocytes are largely free of endogenous receptors that could interfere with the signals of exogenously expressed channels/receptors. Thus, oocytes have been extensively used to characterize the biophysical and pharmacological properties of nAChRs. They have also been used to study the stoichiometry of receptor subunits, the contribution of different subunits to the properties of receptors, and the structure-function relationships with various ligands. For most nAChRs, oocytes have worked extremely well as an expression host [35], [36], [37]. However, in some instances cRNA-injected oocytes have failed to yield readily detectable I_ACh_. For instance, human α9 cRNA-injected oocytes have only small I_ACh_ compared to oocytes injected with its rat counterpart [38], [39]. There is no report to date of successful functional expression of human α9-containing receptors in mammalian cell lines and few reports of successful transfection of rat a9-containing receptors [40], [41].

The article "Functional Expression of Human α9* Nicotinic Acetylcholine Receptors in X. laevis Oocytes Is Dependent on the α9 Subunit 5′ UTR" was published in 2013. Journal: PLoS One.

The translational efficiency of nAChRs in oocytes is influenced by the structure of the injected cRNA [42], [43] including the Kozak sequence [44], the secondary structure [45], [46] and composition of untranslated regions [47], [48]. The 5′ leader sequence preceding the coding region plays an important role in the binding of cap-binding proteins and in facilitation of translation initiation [49]. One approach to improve the translation in oocytes is to flank the gene-encoding sequence with the untranslated regions of highly translatable proteins of *X. laevis*, such as β-globin [50], [51]. When 5′ and 3′untranslated regions (UTRs) of human interferon-β mRNA are replaced by those of *X. laevis* β-globin mRNA, the translation is increased as much as 20- and 300- fold in reticulocyte lysates and in *X. laevis* oocytes, respectively [52]. The *X. laevis* β-globin leader sequence exerts its facilitatory effect presumably by increasing translation initiation, and not by increasing the binding of limiting factors [50]. However, for human α9, the addition of the *X. laevis* β-globin sequence to the 5′ and 3′ UTRs is not sufficient to produce high expression levels.

In this report, we show that the human α9 subunit is the limiting factor in the expression of human α9α10 nAChRs in *X. laevis* oocytes. Furthermore, we found that this expression can be substantially improved by the insertion of the 5′ leader sequence of alfalfa mosaic virus RNA4 (AMV) to the human α9 5′ UTR.

## Materials and Methods

### Ethics Statement

Isolation of oocytes from *X.laevis* frogs was performed in accordance with and under approval of the Institutional Animal Care and Use Committee of the University of Utah.

### cDNA constructs

cDNAs encoding α9 and α10 nAChR subunits from rat were provided by A. B. Elgoyhen (University of Buenos Aires, Argentina). The rat α9 cDNA was in a pGEMHE [51] vector between SmaI and EcoRI restriction sites, and the rat α10 cDNA was in a pSGEM vector (a modified pGEMHE vector) between EcoRI and XhoI restriction sites. cDNAs encoding human α9 and human α10 subunits, in the pGEM-11Zf(+) vector, were generously provided by L. Lustig (University of California San Francisco, San Francisco, CA). The cDNAs encoding human subunits were subsequently inserted into the pSGEM vector between EcoRI and XhoI restriction sites. The oligonucleotides encoding the 5′leader sequence of alfalfa mosaic virus RNA4 (AMV) were synthesized at the University of Utah core facility. The sequence of the synthesized oligonucleotides was as follows: sense- 5′ GGGTTTTTATTTTTAATTTTCTTTCAAATACTTCCACCG 3′; antisense-5′ AATTCGGTGGAAGTATTTGAAAGAAAATTAAAAATAAAAACCCGC 3′. The oligonucleotides were diluted in 10 mM Tris-Cl, pH 8.5 to a final concentration of 107 µM for sense oligonucleotide and 80 µM for antisense oligonucleotide. 20 µL of each oligonucleotide was mixed in an annealing reaction tube. The annealing reaction was as follows: exposure to 95°C for 10 minutes followed by cooling to 25°C over a period of 45 minutes. The annealed oligonucleotide was ligated into MCS of pSGEM vector between the SacII and EcoRI restriction sites.

The article "Functional Expression of Human α9* Nicotinic Acetylcholine Receptors in X. laevis Oocytes Is Dependent on the α9 Subunit 5′ UTR" was published in 2013. Journal: PLoS One.

### cRNA synthesis

The NheI enzyme was used to linearize the vector encoding human α9 and human α10 subunits. *In vitro* transcription was performed using the mMessage mMachine T7 kit (Ambion, Austin, TX). The reaction was followed by DNase treatment. The cRNA was purified with a Qiagen RNeasy kit (Qiagen, Valencia, CA, USA). The cRNA concentration was determined by measuring absorbance at 260 nm on an Epoch spectrophotometer.

### Oocyte isolation and injection

The isolation of the oocytes was performed as previously described [53]. Briefly, stage IV–V oocytes were isolated from anesthetized adult frog. The oocytes were kept at 17°C in ND96 (96 mM NaCl, 1.8 mM CaCl2, 2.0 mM KCl, 1.0 mM MgCl2, 5 mM HEPES, pH 7.1–7.5) supplemented with antibiotics (50 U/mL penicillin, 50 µg/mL streptomycin, 50 µg/mL gentamicin). The oocytes were injected with 50.6 nL of cRNA and incubated for 1–3 days before recording. The amount of cRNA injected into each oocyte varied in different experiments. To compare levels of expression of human and rat α9α10 receptors, 3.3 ng cRNA of each nAChR subunit was injected into individual oocytes. To compare the level of expression of human receptors formed from subunits injected at different ratios, 4.4 ng cRNA of each nAChR subunit was injected into individual oocytes when a ratio of (1) is indicated and 22 ng cRNA was injected when a ratio of (5) is indicated. For all other experiments, 14.4–32 ng cRNA of each subunit was injected.

The article "Functional Expression of Human α9* Nicotinic Acetylcholine Receptors in X. laevis Oocytes Is Dependent on the α9 Subunit 5′ UTR" was published in 2013. Journal: PLoS One.

### Two-electrode voltage clamp recording

ACh-gated currents were recorded from oocytes as previously described [53]. Briefly, an oocyte was placed in ∼30 µL chamber (4 mm diameter ×2 mm deep) fabricated from Sylgard and gravity-perfused with ND96 at a constant flow rate (∼2 mL/min). The oocyte's membrane potential was held at −70 mV using an OC-725B two-electrode voltage clamp amplifier (Warner Instrument Corp., Hamden, CT). To evoke I_ACh_, the perfusion of ND96 was replaced for one-second with ND96 containing100 µM ACh; such a pulse of ACh was applied once per minute. The peak of the ACh-gated current (I_ACh_) was measured and the average of six consecutive I_ACh_ responses served as the control current response.

To minimize potential batch-to-batch variability, oocytes from the same isolation were used to compare the expression of receptors formed from unmodified and modified nAChR subunits. Furthermore, all recordings for a given comparison were performed on the same day.

### Data analysis

Data are expressed as mean ± SEM. Statistical comparisons between two groups were done using Student's t-tests, and those between multiple groups were done using ANOVA test with Tukey's post-hoc comparison.

## Results

### Human α9α10 nAChRs express poorly in X. laevis oocytes

Previous investigations of human and rat α9-containing receptors reported difficulties in the expression of human α9-containing receptors [38], [39]. Consistent with these reports, when cRNAs encoding human α9 and human α10 subunits of nAChRs were co-injected into oocytes at a 1∶1 molar ratio, 100 µM ACh produced small currents (Fig. 1A top), which on average were 30±3 nA (Fig. 1B). Currents of this low magnitude are difficult to utilize for medium throughput pharmacological testing. In contrast, co-injection of rat α9 and rat α10 subunits yielded large currents (Fig. 1A bottom) with an average amplitude of 8067±1638 nA (Fig. 1B). The difference in functional expression between rat α9α10 and human α9α10 nAChRs might be due to the inefficient translation of the human α9 or human α10 subunit or both, and this was explored in experiments described below.

**Figure 1:** Comparison between the levels of exogenous expression of rat and human α9-containing nAChRs in *X. laevis* oocytes. ACh-gated currents were measured in voltage-clamped oocytes as described in Methods. (A) Representative traces from an oocyte injected with human α9 and human α10 cRNA (top) and rat α9 and rat α10 cRNA (bottom). Robust currents were observed with rat cRNA; but only small currents were observed with human cRNA. (B) Comparison of the averaged current responses evoked by 100 µM ACh applications from oocytes expressing human α9α10 and rat α9α10 receptors. The mean current amplitude was 30±3 nA (n = 7 oocytes) for human α9α10 and 8067±1638 nA (n = 7) for rat α9α10, p<0.005. Error bars indicate SEM.

The article "Functional Expression of Human α9* Nicotinic Acetylcholine Receptors in X. laevis Oocytes Is Dependent on the α9 Subunit 5′ UTR" was published in 2013. Journal: PLoS One.

### Functional expression of α9 versus α10 subunitsIn order to assess the influence of α9 vs

α10 subunits on the functional expression of α9α10 nAChRs, we injected cRNA encoding subunits from different species (i.e., rat *versus* human) at a 1∶1 ratio. When human α9 was co-expressed with rat α10, the current amplitude was invariably low in all three batches of oocytes tested, averaging from 5±1 nA to 50±15 nA (Fig. 2 and Table 1). When rat α9 was co-expressed with human α10, the current was readily detectable (Fig. 2 and Table 1) and at a level similar to that seen after co-injection of rat α9 with rat α10 subunits (Fig. 1A bottom and Fig. 1B); the average current amplitude ranged between 732±155 nA and 9755±596 nA, depending which of three batches of oocytes was used. There are at least two possible reasons for the low functional expression: A) rat α10 co-expressed with human α9 produced functionally impaired receptors or B) human α9 subunits are not translated efficiently in oocytes.

**Figure 2:** Comparison between the level of expression of human α9/rat α10 (hα9rα10) and rat α9/human α10 (rα9hα10) receptors. Receptors assembled from injection of cRNAs encoding subunits from different species have different levels of functional expression. hα9rα10 nAChRs were expressed with low efficiency compared to rα9hα10. Results from three batches of oocytes are shown. All oocytes of a given batch were injected on the same day and recordings performed 2 days later. Values of mean current amplitudes are given in Table 1. **p<0.01. Error bars indicate SEM.

**Table 1:** Comparison of the functional expression of receptors following co-injection of cRNA for subunits of different species.^a^

Oocyte Batch #	Receptor	Mean current amplitude (nA)	SEM	n
1	hα9rα10	5	1	4
1	rα9hα10	732	155	5
2	hα9rα10	21	7	7
2	rα9hα10	8200	774	6
3	hα9rα10	50	15	6
3	rα9hα10	9755	596	6

a Graphical representations of these results are provided in Fig. 2.

### Inefficient translation of the human α9 subunit appears to limit assembly of functional human α9/human α10 receptors

When cRNAs encoding human α9 and human α10 subunits were co-injected at a 1∶1 ratio, the I_ACh_ rarely reached 1 µA with the average response equal to 142±23 nA. Oocytes injected with a 5∶1 ratio had currents averaging 5171±748 nA. Injections at a 1∶5 ratio produced oocytes with low average I_ACh_ amplitude equal to 6.5±3.9 nA (Fig. 3 and Table 2). Thus, more abundant cRNA for the α9 subunit leads to substantially enhanced functional expression of α9α10 nAChRs. This increased functional expression suggests that translation of the human α9 subunit is likely a limiting factor in the assembly of α9α10 receptors.

The article "Functional Expression of Human α9* Nicotinic Acetylcholine Receptors in X. laevis Oocytes Is Dependent on the α9 Subunit 5′ UTR" was published in 2013. Journal: PLoS One.

**Figure 3:** Comparison of functional receptor expression following injection of different ratios of receptor subunit cRNA. Differing subunit ratios of cRNA were injected into oocytes and the resulting levels of expression of functional receptors were compared. Recordings were performed 2 days after injection. The data from oocytes of four different batches were combined to determine the mean current amplitudes. Values are given in Table 2. A one-way ANOVA test with Tukey's post-hoc comparison indicated a significant difference between hα9(1):hα10(1) vs. hα9(5):hα10(1), p<0.001, and between hα9(5):hα10(1) vs. hα9(1):hα10(5), p<0.001. There was no significant difference between hα9(1):hα10(1) and hα9(1):hα10(5), p>0.05.

**Table 2:** Comparison of the functional expression of receptors upon co-injection of different ratios of cRNA for specific subunit.^a^

Receptor	Mean current amplitude (nA)	SEM	n
hα9(1):hα10(1)	142	23	23
hα9(5):hα10(1)	5171	748	21
hα9(1):hα10(5)	6.5	3.9	19

a Graphical representations of these results are provided in Fig. 3.

### AMV insertion and expression of human α9-containing nAChRs

Previous investigators have shown that incorporation of 5′UTR of the *Xenopus laevis* β-globin gene facilitates the *in vitro* translation of different proteins in oocytes and other expression systems [50], [51], [54]. In pGEMHE and pSGEM vectors the 5′ leader sequence of the receptor subunit includes the 5′UTR of *X. laevis* β-globin, restriction sites of the vector's multiple cloning site, and the native 5′UTR of the subunit.

Plant viruses use host translational machinery for replication. RNAs of many plant viruses possess efficient translation enhancers [55] that can be used in order to improve the translation of recombinant proteins or expression of receptors in heterologous systems. Among such enhancers are untranslated regions from different viral RNAs. The 5′UTR from alfalfa mosaic virus RNA4, the 3′UTR of brome mosaic virus and the 5′leader of tobacco mosaic virus were shown to be able to enhance the mRNA translation of foreign proteins [56], [57], [58], [59], [60].

In an attempt to improve the translation of human α9/α10 we modified the 5′leader sequence of human α9 and human α10 subunits by introducing the 5′UTR of RNA4 of alfalfa mosaic virus (AMV) into the multiple cloning site of the pSGEM vector (Fig. 4B) between SacII and EcoRI sites, after the 5′UTR of β-globin and in front of the nAChR subunit.

**Figure 4:** Comparison of the 5′ untranslated regions in human α9, human α10, rat α9, and rat α10 subunits. (A) Native 5′UTRs of subunits are between the restriction site and the start codon. (B) The modifications made to the 5′ untranslated region of human α9 and α10 subunits are shown. The 5′UTR of RNA4 of the alfalfa mosaic virus coat protein was inserted into the multiple cloning site of the pSGEM vector between SacII and EcoRI sites. The subunit-encoding sequence is between the EcoRI and XhoI sites.

The article "Functional Expression of Human α9* Nicotinic Acetylcholine Receptors in X. laevis Oocytes Is Dependent on the α9 Subunit 5′ UTR" was published in 2013. Journal: PLoS One.

The AMV incorporation improved the functional expression of human α9 homomeric receptors by 37- to 101-fold, and the human α9α10 heteromeric receptors by 41- to 250-fold, depending on the batch of oocytes used (Fig. 5 and Tables 3 and 4). Despite the variability in the expression levels of human α9 and α9α10 receptors, which is also commonly observed for other nAChRs, the large improvement in expression was highly reproducible.

**Figure 5:** AMV improves the level of functional expression of α9-containing nAChRs. (A) Representative traces and (B) comparisons of the levels of functional expression of homomeric human α9 receptors encoded by cRNA without (A, top) and with (A, bottom) AMV. The results are from three different batches of oocytes, each isolated from a different frog and recorded on 3^rd^ day after injection, are presented. (C and D) Comparison of the level of expression of heteromeric receptors. Recordings were conducted on the second day after injection. Values for mean current amplitude are shown in Tables 3 and 4. *p<0.05; **p<0.01. Error bars indicate SEM.

**Table 3:** Insertion of AMV improves the expression of human α9 homomeric receptors.^a^

Oocyte Batch #	Receptor	Mean current amplitude (nA)	SEM	n
1	α9	7	4	3
1	α9AMV	268	83	5
2	α9	5	1	5
2	α9AMV	372	52	6
3	α9	8	2	5
3	α9AMV	785	167	10

a Graphical representations of these results are provided in Fig. 5.

**Table 4:** AMV improves the expression of human α9α10 heteromeric receptors.^a^

Oocyte Batch #	Receptor	Mean current amplitude (nA)	SEM	n
1	hα9α10	43	6	5
1	hα9AMVα10AMV	10813	1739	10
2	hα9α10	60	11	5
2	hα9AMVα10AMV	6999	1627	5
3	hα9α10	237	41	8
3	hα9AMVα10AMV	9763	1379	8

a Graphical representations of these results are provided in Fig. 5.

## Discussion

In this study, we determined that the functional expression of human α9 subunits of nAChRs in *X. laevis* oocytes depended on the composition of its 5′untranslated region. By introducing the 5′ leader sequence of alfalfa mosaic virus RNA4 into the multiple cloning site of the pSGEM vector just preceding the coding region of human α9 or α10 subunits, we created a vector that gave ∼70-fold higher expression levels of α9 homomeric receptors and ∼80-fold higher expression levels of α9α10 heteromeric receptors compared to those achieved with unmodified vectors.

The article "Functional Expression of Human α9* Nicotinic Acetylcholine Receptors in X. laevis Oocytes Is Dependent on the α9 Subunit 5′ UTR" was published in 2013. Journal: PLoS One.

Since the early demonstration that mRNA encoding nicotinic receptors from *Torpedo californicus* electric organ could produce functional receptors when it is injected into oocytes of *X. laevis* [61], [62], oocytes have frequently been used as an exogenous expression system to study the pharmacology of nAChRs. In most cases, the receptor subunits assemble into functional receptors [36], [63], [64]. However, sometimes the cRNA injected into oocytes fails to yield functional receptors. For example, when cRNA encoding the α6 subunit is co-injected with cRNA encoding the β2 or β4 subunit, there is little or no detectable ACh-gated current [65]. In our laboratory, the unmodified cRNA of human α9 nAChRs failed to produce functional receptors. Other authors also reported difficulties in expressing human α9-containing nAChRs [38], [39]. The ability of cRNAs of rat α9 and human α10 subunits, but not those of human α9 and rat α10, to form receptors with high levels of functional expression suggests that human α9 is a limiting factor in the assembly of functional receptors.

There are several possible factors that can influence the level of functional expression of nAChRs in the *X. laevis* oocyte system. First, the cRNA composition might prevent or interfere with efficient translation. For example, formation of secondary structures may take place that prevent efficient binding of cap-binding proteins and initiation of translation [44]. The nucleotide sequence just preceding the start codon is important for translation initiation. In eukaryotes, the optimal sequence surrounding the start codon is GCCA/GCCaugG [66]. If the purine at the −3 position is changed to a pyrimidine, the efficiency of translation initiation might be reduced. Second, a high G+C content of mRNA can halt efficient transcription and translation by formation of secondary structures. For example, the gene encoding human acetylcholinesterase (AChE) is highly G+C rich (65%) which results in the formation of a secondary structure in the 5′region [67] that serves as an attenuator of transcription. In addition, two highly homologous and highly G+C-rich genes encoding *Bungarus* and rat acetylcholinesterases have strikingly different rates of transcription with approximately equal translation in oocyte functional tests [68]. The difference in the transcription rate is believed to be determined by the differences in the coding sequences.

The G+C content of human α9 mRNA is 49 % for the gene-coding sequence compared to 51% for rat mRNA. α10 subunits are richer in G+C content with a 65% in the human and 59% in the rat subunit. Thus, the G+C content of human α9 is only slightly lower than its rat counterpart. Based on the relatively equal G+C composition of human and rat α9 mRNAs and high homology in nucleotide sequences of gene-coding regions it is unlikely that G+C content contributes to the low level of functional expression observed from unmodified human α9 subunit in our study.

The article "Functional Expression of Human α9* Nicotinic Acetylcholine Receptors in X. laevis Oocytes Is Dependent on the α9 Subunit 5′ UTR" was published in 2013. Journal: PLoS One.

The UTR is another factor influencing translational efficiency. It was shown to be important for the translation of different proteins in different expression systems. Mutations in the UTR affect the translation of aspartyl protease BACE1 protein and HT3A receptor [69], [70], [71]. When the 5′UTR of BACE1 is present, the protein, but not mRNA, level in transfected HEK293, COS7 and H4 cells is reduced as much as 90%. The inhibitory effect of the 5′UTR is due to the upstream open reading frame (uORF) [69], [71]. Due to their importance, the UTR regions are frequently modified to improve translation. For example, it became a common practice to include 5′- and 3′- UTRs of *Xenopus* β-globin into expression vectors to flank the gene-coding region [51]. UTRs of viruses have also been used to replace native UTRs, which results in improved yields of translated proteins or improved functional expression of receptors. For example, the 5′UTR of tobacco mosaic virus enhances the translation of chloramphenicol acetyltransferase and β-glucuronidase in tobacco mesophyll protoplasts, *E. coli*, and *Xenopus* oocytes [56], [58], [59], [72]. The facilitatory effect of the 5′leader is due to recruitment of eukaryotic initiation factor 4G indirectly via heat shock protein 101 [73].

The alfalfa mosaic virus is an RNA virus consisting of three genomic RNAs and one subgenomic RNA (RNA4). RNA1 and RNA2 encode the replicase proteins P1 and P2, whereas RNA3 encodes viral movement protein (MP). RNA4 is 881-nucleotides long, with a 661-nucleotide long coding sequence that encodes a coat protein required for infectivity and replication of the virus [74]. The 5′UTR of RNA4 is 39-nucleotides long, uracil rich and was shown to be able to improve the translation of foreign proteins. Computer-based structure prediction as well as nuclease-sensitivity analysis indicate the unstructured character of the 5′leader sequence, which can facilitate cap-independent translation initiation [75]. This fact might be relevant if cap-dependent translation initiation of unmodified human α9 subunit is disrupted. The substitution of the native 5′UTR with a 37-base-pair AMV RNA4 leader was shown to improve the translation of several proteins [58], [72]. For example, *in vitro* translation of human interleukin 1β and barley α-amylase improved as much as 35-fold [59]. Also, the introduction of AMV into the 5′leader of GABA_A_ receptors improved the expression of those receptors in *X. laevis* oocytes [72].

The article "Functional Expression of Human α9* Nicotinic Acetylcholine Receptors in X. laevis Oocytes Is Dependent on the α9 Subunit 5′ UTR" was published in 2013. Journal: PLoS One.

The 5′UTRs of human nicotinic receptors may be an important factor for receptor function, considering evidence from other systems suggesting that this region could have the regulatory elements important for translation initiation [69], [76], [77]. Many human nAChR subunits have upstream uATG repeats (uATGs) and upstream open reading frames (uORFs). For example, human α9 has an uORF with a length of 36 codons. uORFs are involved in translational regulation of oncogenes by suppressing the level of translation [78], [79]. It is believed that the uORF causes the small ribosomal subunit to stall and therefore halt translation initiation [80]. How the uORF affects the translation of the α9 subunit is an open question. When cRNAs encoding nicotinic receptor subunits are injected into oocytes at a 1∶1 molar ratio, it is assumed that the two subunits will be translated with equal efficiencies so the amount of protein of the two subunits will also be produced in a 1∶1 ratio. However, different receptor subunits might be translated with different efficiencies.

mRNA stability might be a contributing factor to the observed different levels of expression between unmodified human α9-containing receptors and rat α9-containing receptors. One of the factors that determines the stability of mRNA is located within 3′-end of mRNA. In particular, the poly(A) tail is required to ensure high functional stability of the mRNA as was shown for rabbit globin protein [81], [82]. The 3′UTR of the human α9 subunit had a short (6 nucleotides) native 3′UTR, followed by the 3′ UTR of *Xenopus* β-globin, followed by a poly(A) tail. In contrast, the modified construct incorporated the 5′ UTR of the alfalfa mosaic virus RNA4. This addition may slow degradation of the mRNA.

Another factor that may contributes to the fast turnover of mRNA is an AU-rich region at 3′-untranslated region. Many RNA-binding proteins such as ELAV-like proteins (HuD, Hel-N1, HuC, HuR) bind to AU-rich regions at the 3′-untranslated region of RNA and prevent degradation of mRNA [83]. Human α9 as well as rat α9 subunit 3′UTRs have six non-overlapping AUUUA motifs separated by non-AU nucleotides in a U-poor region. In addition, they have one AAAAUUUAAAA motif.

A second possibility for low expression level of receptors in oocytes is the lack of postrtranslational modifications in the oocyte expression system. The possible posttranslational modifications of nAChRs include proteolytic cleavage, disulfide bond formation, glycosylation, palmitoylation, fatty acid acylation, phosphorylation, amidation, hydroxyprolination, proline isomerization, etc. [84], [85], [86], [87]. The lack of functional expression of α6-containing receptors is likely due to posttranslational mechanisms, insofar as functionality is achieved when the C-terminus of the α6 subunit is replaced with the C-terminus of an α3 subunit implying that important regulatory elements for efficient receptor function are located outside of ligand-binding domain [65].

The article "Functional Expression of Human α9* Nicotinic Acetylcholine Receptors in X. laevis Oocytes Is Dependent on the α9 Subunit 5′ UTR" was published in 2013. Journal: PLoS One.

A third possibility is the lack of appropriate chaperones in oocytes. There are several chaperones described for nicotinic receptors such as BiP, calnexin, Erp57, and RIC3 [88], [89], which facilitate proper folding and improve functional expression of receptors. Nicotine exposure causes an upregulation of nicotinic AChRs in brain as well as *in vitro*, and a possible explanation of this effect is through the chaperoning by nicotine [90], [91], [92]. The RIC-3 is a chaperone that upregulates the expression of α7 nAChRs in oocytes [93], [94], [95], [96]. Interestingly, RIC-3 has no effect on the expression of α9 receptors [40], [97].

There are few reports of successful expression of α9 receptors in mammalian cells [98]. GH4C1 cell line derived from pituitary gland was successfully transfected with rat α9α10 receptors [41]. Here, the average ACh-evoked currents ranged between 16 pA to 300 pA. Also, an α9/HT3a chimera, where the N-terminus of rat α9 was fused to the C-terminus of mouse HT3a receptor, produced functional receptors [99]. Mouse α9α10 receptors were successfully transfected into HEK293 cells [98]. The problem of the lack of expression of human α9 receptor in mammalian cell lines was addressed in several reports [40], [98], [99], [100]. It was shown that co-transfection of human α9 and α10 subunit with AChR-associated proteins rapsyn and chaperone RIC-3 in CL4 cells increased the cytosolic calcium level after application of 100 µACh but no measurements of ionic current from α9-containing receptors were reported [100]. It is still an open question as to whether the lack of functionality in mammalian cells is due to inefficient transcription, translation, improper folding, and lack of chaperoning or posttranslational modifications or a combination of these.

In our current study, we observed the effect of the 5′UTR of the human α9 subunit on the expression of functional receptor. We conclude that the inefficient expression of human α9-containing receptors can be improved by modifying 5′UTR of the cRNA encoding the subunit. It is possible that the initiation codon of the original unmodified subunit is in unfavorable form such that the small ribosomal subunit fails to associate with the RNA. By including the 5′UTR of RNA4 of alfalfa mosaic virus, we were able to construct an RNA, which when expressed in *X. laevis* oocytes, can be used to screen new ligands which bind to the α9* receptor (* denotes possibility of other subunits). The reasons for the poor ability of α9 receptors (both rat and human) to be expressed in the mammalian cells still remain to be explored.

The article "Functional Expression of Human α9* Nicotinic Acetylcholine Receptors in X. laevis Oocytes Is Dependent on the α9 Subunit 5′ UTR" was published in 2013. Journal: PLoS One.

Transcriptional and translational mechanisms are likely involved in regulation of human and rat α9 subunit expression in native tissues. In the rat adrenal medulla expression levels of α9, α3, and α7 subunits were determined by quantitative PCR [19] and the level was lowest for the α9 subunit. However, the same study showed that transcription of α9, but not α3 and α7 subunits, is upregulated in response to stress. Regulation of transcription and translation of nAChRs may also be relevant in the context of smoking. The concentration of nicotine in active smoker plasma can be 100 nM to 1 µM. Chronic exposure to nicotine leads to activation and desensitization of nAChR subtypes including α4β2 and α7. As a result, the level of expression of α4β2 nAChRs is increased in the brain [101]. Smoking is also associated with carcinogenesis, and nicotine-derived metabolites NNK and NNN are considered carcinogenic in lung, breast, and bladder cancers. α9 receptors mediate cell proliferation of breast cancer cells, and increased α9 nAChR subunit mRNA levels were observed in breast tumor tissues [102]. Moreover, α9-nAChR mRNA expression was higher in advanced-stage tumors. It was also shown that nicotine upregulates the mRNA as well as protein level for α9 receptors in breast tumor tissue [102]. The mechanism by which nicotine treatment leads to this upregulation remains elusive. α9 subunit expression seems to be important for cell proliferation, therefore, the mechanisms, whether transcriptional or translational, that control subunit expression might open exciting new avenues for control of tumorigenesis.

Our findings suggest the involvement of 5′-untranslated region in the efficient expression of human α9-containing receptors in oocytes. It remains to be investigated whether 5′untransated region contributes to the regulation of translation of α9 subunit *in vivo*.
